# Innovative Practice of Music Education in the Universities in the Context of 5G Network

**DOI:** 10.1155/2022/3451422

**Published:** 2022-06-14

**Authors:** Shaohan Huang

**Affiliations:** College of Contemporary Music, Yango University, Fuzhou, Fujian 350015, China

## Abstract

Music education is among the most significant subjects covered in providing high-quality education in Chinese universities and colleges. Music education is critical to providing high-quality education to students. It contributes significantly to the development of students' creative motivation, inventive capacity, and personality development. Music education provides excellent outcomes in music instruction and fosters students' original thinking and comprehensive abilities, and therefore supports the overall development of high-quality education. With the development of the educational system, it is becoming more vital to teach students a high level of musical literacy. With the advent of 5G mobile communication, it will become one of the core technologies in Chinese music education, providing an innovative framework for music education. In this study, a novel music education model is proposed for the development of music education using the GTZAN dataset which is comprised of 100 distinct specimens for every genre and ten various kinds of music. The dataset is normalized to prepare it for further processing and the characteristics of the song are retrieved using a technique called spectrum-based feature extraction (SBF). Bi-recurrent neural networks (Bi-RNN). are used to classify objects in space. An improved TCP congestion control algorithm (ITCCA) is proposed for efficient data transmission between the 5G networks. To optimize the performance of the transmission protocol, the honey bee optimization algorithm is employed. The performance of the proposed model is examined and contrasted with that of the currently used approaches. The proposed model shows high performance in terms of throughput, average delay, and packet delivery ratio. The model has the potential to successfully integrate 5G technologies and music education and provide the students with rich and diversified teaching materials and flexible instructional formats.

## 1. Introduction

A significant push has been given for contemporary teacher learning by current scientific and technical discoveries, particularly the rapid growth of computer technology as represented by “music education + 5G.” Modern curriculum reform has pushed the bar for teachers' ability to teach to new levels, resulting in increased expectations for them [1]. Traditionally, education has been delivered via schools, and individuals have only had a few options for learning. However, as “Music education + 5G” continues to develop, more channels and methods of disseminating knowledge are becoming available, and the methods of education have been altered significantly. In recent years, the continual growth and strengthening of “Music education + 5G” has steadily eroded the stronghold of schools on information distribution, facilitating the shift from a limited to an accessible educational system. When “Music education + 5G” is developed, people will receive education on campus and the 5G platform in the future [2]. As a result, the positive growth trend of actual learning, complementing, and expanding online education will be realized. Music education and 5G are currently being developed and the overall development trend is positive. With the ongoing growth of “Music education + 5G,” so far, new types of music training, including catechism, mobile applications, have helped to provide the groundwork for future growth and research in music education [3].

It is expected that 5G technology, also known as next-generation mobile cellular technologies, will significantly impact our every day in the near future. The introduction of 5G will bring about significant improvements in present network technologies in terms of increased capacity, more dependable service, and a greater density of devices [4]. Because of their unique qualities, these features can affect or even change a wide variety of human activities, from business to entertainment, by improving presently accessible services and introducing whole new ones. This will be possible through the enhancement of current services offered and the initiation of entirely new services. Therefore, it is believed that 5G will influence educational experiences as well. In music education, a lot of bandwidth is critical for exchanging high-quality multimedia streams and it is essential to keep latency in bidirectional connection to a minimum, ideally, in the millisecond range [5]. During the Fifth Mobile 5G Expo in China, the concept of “5G + music education” was introduced to integrate 5G as a source with all walks of life, boldly innovating and promoting the fast growth of China's economy benefiting people via this platform. “5G Plus” is a hub that unites people from all areas of life via network information and communication technology, which establishes a new field and allows for new developments in that sector [6].

With the arrival of the 5G era, 5G mobile communication will play a significant role in our future education, and 5G technology will become one of the most important educational technologies. 5G can connect music teachers with their students while also allowing new music technologies like virtual reality, augmented reality, and improved streaming. Students may take part in events even if they cannot make it in person, and they can immerse themselves more fully in the artists' vision by employing multiple camera angles and virtual environments created to match the music.

In this study, a new music education model is presented for the development of music education using the GTZAN dataset. The dataset is preprocessed and the discriminant features of the songs are retrieved using the spectrum-based feature extraction method. Bi-recurrent neural networks are used to classify objects in space and an improved TCP congestion control algorithm is employed for fast data transmission between the 5G networks. To optimize the performance of the transmission protocol, the honey bee optimization algorithm is utilized.

The rest of the manuscript is organized as Section 2 illustrates the related works in the field of 5G and music education. In Section 3, a detailed description of the proposed bi-RNN algorithm and honey bee optimization technique are presented.  Section 4 is about performance analysis and the conclusion is given in Section 5.

## 2. Related Work

The Internet is used in all fields of education, learning, and life. Many new music teaching models have emerged through the Internet platform and information and communication technologies. Many scholars have presented advanced models for the development of music education. Barate et al [7] employed virtual reality and augmented reality technology-based activities to outline the major features of 5G and proposed an application in music education as an example. The authors in [8] used multimedia networked communications to communicate with professors and students and provide the course's contents and recommended that the development of modern distant education is essential for developing a lifelong learning system for individuals in the information age. Law and Hou [9] examined the legitimacy of values in music education to prepare students for admission into China's new “knowledge society” and illustrated how values education connects to the teaching of musical and nonmusical meanings in the twin contexts of nationalism and globalization and some of the difficulties that value education encounters in school music classes. Zhang [10] worked on the Chinese ethnic minority's musical and cultural traditions in government-designed national K1–9 music textbooks. To realize speech and music recognition, this work applied the distinct principles of the magnitude of new information in the signal sequence of speech and music, as well as their changing range, to accomplish the intended effect. Lin [11] investigated the importance of assessing music teaching ability before summarizing the use of neural network and deep learning technologies in music teaching ability evaluation and created an assessment model using a compensating fuzzy neural network technique and tested its correctness. In [12], a power iteration-based technique of system resource allocation for 5G music education is proposed. The unloading system's throughput is defined as an optimization challenge, with the best allocation of regular power achieved via an iterative method of the optimal solution. A heterogeneous network that depends on network edge is constructed to compensate for edge servers' loss efficiency and resource consumption to discover the best technique for ensuring the Nash equilibrium point. Sun [13] used multidimensional connection feature fusion and clustering algorithms to present an optimal fusion approach for an “offline and online” mixed music education model in the context of 5G. The author in [14] provided a historical overview of popular music in China throughout the twentieth century, both in the community and in school music, and examined how, since the beginning of 2000, reforms in music education have included popular songs into the curriculum. The developed system is divided into three sections: the multiple data mechanism, the server manager module, and the database administration module [14]. The genetic algorithm is used to integrate the data after the synchronization multimodal voice learning data are processed by the synchronized multimodal vocal education information processing [15]. As a result of mixing big data with customized recommendation algorithms based on the collaborative filtering recommendation system, a hybrid recommendation algorithm is developed (CF).

To acquire the user assessment matrix, a large amount of data are required. Li [16] used the Pearson correlation coefficient to determine user similarity and constructed the closest neighbor set, the *k* nearest set of target users, and the subscriber recommendations set. As a part of this process, a questionnaire was created to gather the actual assessment ratings of each user on the audio contents. Cao [1] examined the possibility of using 5G for music education with big data and in light of rapid scientific and technological improvement, to clarify and lead music teachers to use spontaneous and conscious awareness of new media and fully apply new science and technology in the information society for future music classroom teaching, and to inspect the mode, method, trend, characteristics, advantages, and disadvantages of using 5G for music education. Although many researchers and analysts have investigated the role of 5G in the development of music education, the application of 5G communication technologies in the music field is still in its infancy and requires in-depth investigation and improvement. This study presents a 5G music education model using machine learning to classify musical sounds and an improved TCP congestion control algorithm is presented for fast data transmission between the 5G networks.

## 3. Proposed Work

The introduction of the 5G network in education will result in a significant change in music education [17]. Compared to the existing network technologies, 5G will provide considerable gains in terms of bandwidth, service dependability, and device density. Furthermore, this study focus on music education, a field in which having a huge network capacity is vital for sharing high-quality multimedia streams, and two-way communication latencies should be maintained within the milliseconds' range. A simplified illustration of the proposed technique is shown in Figure 1.

### 3.1. Dataset

In this study, the GTZAN dataset is used since it has been used in much earlier research and would enable us to assess the model more correctly. The dataset of GTZAN contains 100 distinct specimens for every genre, and ten various kinds of music are used [18]. Since the input data have not been processed, it may contain duplicated sequences and incomplete data. An in-depth cleaning and high-level processing have been performed to remove recurring and duplicate occurrences, as well as missing data. Because of the large number of features in this database, approaches for extracting features are required to exclude characteristics that are not important. During the preprocessing stage, the dataset is normalized. (1) describes how the s-score is generated in the first step of the normalizing.

(1) $$\begin{array}{c} U=\frac{Tu-\omega }{\alpha }, \end{array}$$

where *ω* is the mean, *α* is the standard deviation, then the *U* can be written as follows:

(2) $$\begin{array}{c} U=\frac{Tu-\overset{-}{Tu}}{UUK}, \end{array}$$

where $\overset{--}{Tu}$ of the sample is mean and *UUK* is the standard deviation of the samples.

The randomized sample is made up of the following individuals:

(3) $$\begin{array}{c} U_{a}=\beta_{0}+\beta_{1}Tu_{a}+\varepsilon o_{a}, \end{array}$$

where *εo*_*a*_ represents the error that depends on *α*^2^

Next, the errors must be independent of each other and as indicated in the following section.

(4) $$\begin{array}{c} \frac{\sqrt{v}}{t_{a}}\frac{t}{\sqrt{t^{2}+v-1}}, \end{array}$$

where *t*_*i*_ is the random variable.

In the next step, the standard deviation is used to normalize the variations in the variables. It is possible to estimate the moment scaling deviation by using the given equations:

(5) $$\begin{array}{c} \text{FUK}=\frac{\lambda^{\text{fuc}}}{\theta^{\text{fuc}}}, \end{array}$$

where *fuc* denotes a scaling moment.

(6) $$\begin{array}{c} \lambda^{\text{fuc}}=\text{Exp}\left(Ti-\alpha \right)\wedge \text{FUC}, \end{array}$$

where Exp represents the expected value and *Ti* represent a random variable.

(7) $$\begin{array}{c} \theta^{\text{fuc}}=\sqrt{\text{Exp}\left(Ta-\alpha \right)}\wedge \text{FUC}\wedge 2,\\ t_{c}=\frac{\text{fuc}}{Ta}, \end{array}$$

where it is the coefficient of variance.

By changing the values of all parameters to 0 or 1, the feature scaling process is completed. The following method is used to accomplish the normalization.

(8) $$\begin{array}{c} T_{i}=\frac{t-t_{\min}}{t_{\max}-t_{\min}}. \end{array}$$

The data range and irregularity of the input may remain unchanged after it has been normalized. To reduce delay, this step is completed. Next, the normalized data may be utilized as an input to the following phases in the procedure.

### 3.2. Spectrum-Based Feature Extraction

#### 3.2.1. Centroid of the Spectral Spectrum

Spectral centroid (also known as the frequency spectrum centroid) is a statistic used in digital signal processing to describe the frequency band. It has a close link with the intensity of the noise source[19]. Since the spectral centroid better represents the brightness of the sound, it is based on digital audio and musical signal analysis. It is a tool for evaluating music's timbre. It is a musical term. Mathematically, it can be defined as follows:

(9) $$\begin{array}{c} D_{s}=\frac{\sum_{a=1}^{A}B_{s}\left[a\right]*a}{\sum_{a=1}^{A}B_{s}\left[a\right]}, \end{array}$$

where letter ‘a' designates the location of the “centroid” of the frequency range. It is closely related to the intensity of the noise source. The term *B*_*s*_[a] designates the Fourier transform magnitude.

#### 3.2.2. Flux Spectral

The flux spectral is a broad term that refers to the pace at which the signal spectrum changes [19]. It is determined by calculating the current frame spectrum to the range of the previous frame. The 2-norm among two normalized spectra is often used to compute it, which is more exact. The spectrum flux computed in this method does not depend on the period since the spectrum has been normalized. To compare two signals, their amplitudes need to be known. It is a common practice to employ flux spectral to identify the timbre of an audio source or whether or not to pronounce it. The flux spectral can be computed as follows:

(10) $$\begin{array}{c} U_{s}=\sum_{a=1}^{A}\left(A_{s}\left[a\right]-A_{s-1}\left[a\right]\right). \end{array}$$

#### 3.2.3. Contrast in the Spectral Range

Spectral contrast is a property that is used to categorize different types of music [20]. Spectral contrast is described as the variation in decibels (DB) between both the ridges and valleys of a frequency range, which may illustrate the relative spectral features of different types of music and sounds.

#### 3.2.4. Cepstral Coefficients at Mel-Scale Frequencies

Because the ear cochlea contains filtering qualities, it may map various frequencies to different places on the basilar membrane, which allows for more accurate mapping. As a result, the cochlea is often referred to as a filter bank [21]. Psychologists were able to acquire a set of filter banks comparable to the cochlear effect via psychological research, which they named the Mel frequency filter bank, based on this characteristic. Because the sound level experienced by the human ear is not linearly proportional to the frequency of the sound, researchers have developed a new notion known as Mel frequency to account for this. The Mel frequency scale is better following the acoustic qualities of the human ear than the Richter frequency scale. The following is the relationship between Mel frequency and the integer u:

(11) $$\begin{array}{c} \mu_{\text{mel}}=25955g\left(1+\frac{u}{700}\right), \end{array}$$

where *μ*_mel_ denotes the Mel frequency conversion and *u* denotes the frequency.

For starters, the audio signal is separated into frames and pre-emphasized before being windowed. After that, a short-time Fourier transform is conducted to acquire the frequency spectrum of the audio signal. Next, we set the Mel–frequency bank of the *L* channel to the Mel frequency by adjusting the Mel filter bank of *L* stations. The *N* value is calculated when the signal has reached its most significant frequency, which is usually between 12 and 16. Each Mel filter has the same spacing on the Mel frequency as the previous one. (12) computes the relationship between the three frequencies of neighboring triangle filters:

(12) $$\begin{array}{c} d\left(l\right)=h\left(l-1\right)=0\left(l+1\right). \end{array}$$

Assuming that *d* (*l*) denotes center frequencies, *h* (*l*) denotes the upper frequency's limit, and *o* (*l*) denotes lower frequency's limit.

The outputs of the filter that get through the Mel filter are as follows:

(13) $$\begin{array}{c} y\left(l\right)=\sum_{k=o\left(l\right)}^{h\left(l\right)}\frac{V_{l}\left(k\right)}{X_{b}\left(k\right)},l=1,2,\ldots N. \end{array}$$

The filter's frequency characteristics are as follows:

(14) $$\begin{array}{c} v_{l}\left(k\right)=\left\{\begin{array}{c} \frac{k-o\left(l\right)}{\left(\left(l\right)-o9l\right)},o\left(l\right)\leq k\leq \text{d}\left(l\right)\\ \frac{h\left(l\right)-k}{h\left(l\right)-c\left(l\right)},c\left(l\right)\leq k\leq h\left(l\right) \end{array}\right\}, \end{array}$$

The discrete cosine is transformed to MFCC by taking the natural log of the filter's actual output. This is computed as follows:

(15) $$\begin{array}{c} {\text{MFCC}}_{\text{MFCC}}\left(a\right)=\sum_{l=1}^{L}\mathrm{lg}y\left(l\right)*\;\cos\left[\pi \left(l-0,5\right)\frac{a}{L}\right],\\ a=1,2,3\ldots N. \end{array}$$

#### 3.2.5. Classification Using the Bi-RNN (Recurrent Neural Network)

Over time, the RNN may detect the inherent structure buried in the sequence. The audio signal may be thought of as a time sequence in and of itself. The spatial dependency of the audio signal in the time dimension may be captured by using the RNN to process music. In the temporal dimension, the sound spectrum is likewise widened. Because the feature map after one-dimensional convolution can be thought of as a temporal feature sequence, the usage of the RNN to analyze sound spectrum information may also be considered in this way [18]. This research employs the Bi-RNN to describe the music sequence to better represent the multidirectional dependency in the time dimension and get closer to the brain's perception of music. The Bi-RNN takes into account both the previous and subsequent inputs, which may aid with data modeling. The architecture of the Bi-RNN is shown in Figure 2.

In the estimate of the future, $\overset{⟶}{z^{a}}$ is connected to, and in $\overset{⟶}{z^{a-1}}$ and in computation in reverse, is $\overset{⟶}{z^{a}}$ connected to $\overset{\leftarrow }{Z^{a+1}}$ and $\overset{⟶}{z^{a}}$ indicates the hidden layer's current condition. The calculating formula is as follows:

(16) $$\begin{array}{c} {\overset{\leftarrow }{Z}}^{a}=u{\left(X^{xa}+M\right)}^{\overset{\leftarrow }{Z}+1}. \end{array}$$

To get the final network output, we combine the forward and rear of each network step.

(17) $$\begin{array}{c} T_{a}=M\overset{\leftarrow }{z^{a}}+M^{\prime }\overset{⟶}{z^{a}}. \end{array}$$

#### 3.2.6. Improved TCP Congestion Control Algorithm

Live broadcasts would be out of place with this protocol designed for on-demand access to an extensive music collection. If a customer wants to upload a song, they will need to have the whole track on their computer. So, it simplifies things by not indicating which portions of a track a client owns anymore. The drawbacks are minimized due to the small size of the tracks. Instead of using UDP, which is the most common streaming app transport protocol, Spotify uses TCP. To begin with, having a dependable transportation protocol makes protocol plans easy to implement. Second, TCP is suitable for the network because congestion management is favorable, and stateful firewalls benefit from explicit relationship signaling. Finally, since streamed content is shared through a mentoring network, resending missing packets is beneficial to the program [22]. A single TCP connection is utilized between two hosts, and messages are multiplexed via the protocol specification. A client maintains a TCP connection to a Spotify server while it is active. Priority-ordered is buffering and sorting application layer messages before being delivered to the operating system's TCP buffers. Messages required to allow interactive surfing, for example, are prioritized above bulk traffic.

#### 3.2.7. Honey Bee Optimization Algorithm

For both functional and combinatorial optimizations, the honey bee's method uses random search and neighborhood search. The fundamental goal of this method, as illustrated in Figure 3, is to identify an optimum solution using honey bees' natural foraging activity. In general, scout bees (*n*), chosen sites in visited websites (*m*), resting criterion, best places in sample locations (*e*), starting patch size, which includes the network's size and its surroundings, bees for selected sites, and bees for sites are needed. The fitness of bees is assessed after they are randomly put in an area. The honeybees with the best fitness levels are chosen, and the bees who visit the places are selected for the neighborhood search. Now, it is time to recruit bees and assess their fitness at the desired locations. The fittest bees from each patch are chosen. The fitness of the remaining bees is evaluated after they are allocated to a search area at random. The stages are then repeated until the condition for halting is fulfilled. The bees method is utilized in various applications, including clustering techniques, neural network pattern matching, and construction. In sensors, nodes near the sink must transfer their data and data received nodes further away, depleting the energy of nodes near the sink. The network isolation issue, also known as the HOT SPOT problem, is caused by the surrounding nodes' energy depletion. It will significantly alleviate this issue, if sink mobility is used since the energy consumption of neighboring nodes will be balanced. In this study, biological methods are also utilized to improve the packet delivery ratio, throughput, and delay.

## 4. Performance Analysis

### 4.1. Music Performance

In this section, we analyze the performance of the proposed method and compare it with existing methods.  Figure 4, 4(a)–4(d) shows that the real data and simulated data curves agree, indicating a good model fit. The amount of negative emotion decreases, whereas the neutral and positive mood indexes increase, showing that the population is less suspicious and concerned than when “Music education + 5G” was initially introduced after a year of practice and investigation. 5G users started to think more critically about the issues that arose throughout the “Music education + 5G” process, and they expressed a favorable attitude toward “Music education + 5G” and a more accurate description.

Figure 5 demonstrates that pop music is more popular among college students because it is closer to their lives. However, there are plenty of students who like classical, instrumental, and traditional music. The majority of pupils have a rudimentary understanding of music and can read pentatonic and short scores, and they learn music and associated basic information via many methods.

Figure 6 shows that 71.14% of students feel that music electives are required, while just 5.67% say they are not, and the remainder are undecided. This is because the majority of pupils feel that music education may help them develop emotion and control their mood (55.20% and 39.28%, correspondingly), as well as the fact that music education may aid in the development of intellect, provide entertainment, and improve life (35.16%). Students fully comprehend and agree with the uses and benefits of music, yet many have qualms about music's various learning activities at school.

On the one hand, as shown in Figure 7, universities are increasingly focusing on 5G music education and introducing new music classes and actions; however, due to a lack of publicity, the 5G music teaching method is not well known, and educators' overall participation is low, resulting in the majority of students not participating in school music activities.

### 4.2. Network Performance

#### 4.2.1. Throughput

The throughput is defined as the number of data packets received by the destination at a certain time.  Figure 8 shows the throughput comparison between the present and proposed methods. We compared the throughput of the proposed system with that of TCP [19], SACK [20] TCP vegas[21], and SCTP [23]. The graph clearly shows that the recommended strategy has a higher throughput of 700 for 80 nodes than traditional techniques.

#### 4.2.2. Average Delay

It is the amount of time that it takes a packet to travel from its origin to its destinations.  Figure 9 depicts a side-by-side comparison of the average delay for the present and proposed techniques. We compared the average delay of the proposed system with that of TCP [19], SACK [20] TCP vegas [21], and SCTP [23]. The graph shows that the suggested process transmits data with the least latency compared to conventional methods.

#### 4.2.3. Average Packet Delivery Ratio

It is calculated by dividing the obtained data packets by the transmitted data packets and is used to determine routing effectiveness. The comparison of packet delivery ratios for the proposed and existing methods is shown in Figure 10. The average packet delivery ratio of the proposed system is compared with that of TCP [19], SACK [20] TCP vegas [21], and SCTP [23]. It is evident that the proposed technique has a higher average packet delivery ratio than the existing methods which confirms the superiority of the proposed method.

## 5. Conclusion

The Internet is used in all aspects of our lives, including learning, education, and entertainment. Through the Internet platform and information and communication technology, many new models of education have evolved. With the arrival of high-speed Internet and 5G, all disciplines will undergo an unprecedented shift. This study employed the GTZAN dataset, which contains 100 individual specimens for each genre and ten different forms of music, to propose a new music education model for the advancement of music education. The dataset was normalized, and the song's features were extracted using a technique called spectrum-based feature extraction. To classify objects in space, a machine learning algorithm called bi-recurrent neural networks was used. For effective data transfer between 5G networks, an improved TCP congestion control algorithm (ITCCA) was employed and the honey bee optimization algorithm was used to improve the transmission protocol's performance. The proposed model showed high performance in terms of throughput, average delay, and packet delivery ratio as compared to the existing models. The model can successfully combine 5G technology with music education, as well as provide students with a wide range of teaching materials.

## Figures and Tables

**Figure 1:** Schematic representation of the proposed flow work.

**Figure 2:** Architecture of the Bi-RNN.

**Figure 3:** . Honey bee optimization.

**Figure 4:** (a,b,c,d) Constantly shifting hot index of music education + 5G. (a) In the beginning. (b) After a period of time. (c) Later. (d) Now.

**Figure 5:** Different types of music.

**Figure 6:** Different types of music education in 5G.

**Figure 7:** 5G music education satisfaction level.

**Figure 8:** Throughput vs. number of nodes.

**Figure 9:** Average delay vs. number of nodes.

**Figure 10:** Average packet delivery ratio vs. number of nodes.

## Data Availability

The data underlying the results presented in the study are available within the manuscript.
